# A Study on the Effects of Chinese Massage on Physical and Mental Health in Participants Based Smart Healthcare

This article has been retracted.

**DOI:** 10.1155/2022/9732355

**Published:** 2022-01-07

**Authors:** Ko-Hsin Chang, Chih-Hsiang Hung, Tzu-Yun Lin, Hsiao-Hsien Lin, Yi-Ling Chen

**Affiliations:** ^1^Department of Physical Education, Chinese Culture University, Taipei 11114, Taiwan; ^2^Center for General Education, Taipei Medical University, Taipei 11045, Taiwan; ^3^Department of Sport Information and Communication, National Taiwan University of Sport, Taichung City 404401, Taiwan; ^4^School of Physical Education, Jiaying University, 514015 Meizhou City, Guangdong Province, China; ^5^Department of Sports Medicine, China Medical University, Taichung, Taiwan

## Abstract

The purpose of this study is to understand the influence of the effect of the smart Chinese massage appliance on the participants' sports performance and physical and mental health after intermittent exercises. The study was performed by a mixed-study method. First, the experimental research method was used to design an experimental procedure and specifications such as data collection scope. Next, the quantitative research was carried out, using SPSS 26.0 statistical software to analyze data from the questionnaire. Then, the qualitative research was carried out by interviewing experts and respondents and obtaining their opinions. Finally, all the data were collated and analyzed using the multidimensional review method. *Findings*. Chinese massage significantly improved the physical fitness, exercise performance, body composition, and physical and mental health status of high-strength cyclic exercise participants. High-strength exercises can improve the physical and mental health of men. Medium-strength exercises could improve current conditions for women. Oxygen intake remained peaked for 8 sessions for men and increased after 30 sessions for women. Both groups required a 1-2-week adaptation period but had different exercise performance periods. After the experiment, head and back pain, as well as stress and negative emotions, was improved. The high intensity of the exercises relieved fear, headache or head stress, overeating, and other problems.

## 1. Introduction

With the advancement of science and technology, electronic software facilities or information is flooded, which has changed human behavior and daily life. The willingness of the population to go out and exercise is decreasing, and youth and children in countries around the world are affected by the lockdown policy [1]. Their behaviors and lifestyles are changing, with less physical activity and more sedentary or lying-down time. This phenomenon will accelerate the deterioration of adolescents' physical and mental health [2], decreasing cardiorespiratory and physical adaptability, increasing body weight [3], reducing social and interpersonal interactions, increasing psychological stress [4], and even diminishing the willingness to work or study [5], and this phenomenon may extend into adulthood [6]. Globally, more than 70% of adolescents have low levels of physical inactivity and inadequate adaptive capacity [7]. Governments and scholars are concerned that this phenomenon will worsen [1], affecting youth growth and overall national development.

Although the improvement of physical and mental health can start with exercise [8], most students are affected by personal spatial and physical barriers [9], as well as internal and external factors such as location, time, and cost that limit university students' participation in exercise [10]. Therefore, finding time-saving, effective, and easy-to-operate exercise modalities to provide university students with options to engage in exercise and improve their physical and mental health status will be the most urgent issue at present. The intermittent cycle exercise method features short time consumption and high efficiency [11], which breaks from the conventional method of long-duration and low-strength aerobic exercise for fat loss [12]. The intermittent cyclic exercise mode can be divided into high-intensity (HICT) and moderate-intensity (MICT) according to the difference in intensity. While studies have found that HICT is more effective in improving mental and physical health and physical fitness, both modes are effective in improving cardiorespiratory fitness in healthy adults [13]. However, studies have shown that although intermittent cyclic exercise has a significant effect on participants' exercise performance, it is associated with periodic exercise performance due to postexercise fatigue and short-term deterioration of muscle strength [6, 14, 15], which affects physical and mental health [16]. Therefore, if no attention is paid to the phenomenon of exercise fatigue by immediately taking exercise or fatigue relief measures to restore health, the level of fatigue will exacerbate resulting in qualitative changes. This will affect the willingness of university students to continue to exercise and perform in sports [17], interrupting their plans and effectiveness in improving their physical and mental health. It is a disturbance and a hindrance for university students who want to improve their physical and mental health through exercise.

Tuina is one of the methods of treatment and physical care from ancient China [18], of which massage is one of the techniques [19]. It can effectively relieve muscle tension, alleviate cardiovascular and visual disorders, and improve overall body quality [20]. With the prevalence of sports and healthcare, the application of massage in sports has been gradually established [21]. In fact, the current research topics on the application of sports massage techniques to muscle injury have gradually become more refined [22, 23]. However, researchers have found that although scholars around the world are becoming aware of the impact of the COVID-19 epidemic on the health of the population [24–26], little attention has been paid to the status of the subjects who have continued to exercise [27]. Moreover, there are few studies on the topic of intermittent cyclic exercise. Very few studies have explored the effects of Chinese Tuina on the adaptability, performance, and physical and mental health of university students participating in the intermittent exercise. Studies on the application and effects of intermittent cycles of different intensities have not been found to date either. Therefore, the investigators believed that, during the current situation of the COVID-19 epidemic, applying the Chinese massage to university students participating in intermittent exercise of different intensity and investigating their adaptive capacity, athletic performance, and physical and mental health effects would help to understand whether Chinese massage could delay or accelerate the recovery of fatigue, enhance physical fitness, and improve body composition as well as physical and mental health in university students adopting intermittent exercise during the epidemic.

## 2. Literature Review

### 2.1. Intermittent Cycle Exercise

The intermittent exercise involves the repetition of multiple exercises for relatively short periods of time [28]. High-strength intermittent exercise is an exercise plan that exceeds the anaerobic threshold intensity or is close to or greater than the maximum oxygen intake intensity [29]. Intermittent cyclic exercise is a kind of exercise pattern that uses different exercise movements with a scheme and purpose to train various muscle groups in the body [29].

Intermittent cycle exercise is a break from the conventional method of long-duration, low-intensity aerobic exercise for fat loss [25]. The 7-minute high-intensity interval exercise (7-minute HICT) emphasizes that it can be performed in a safe environment for participants in any location, without special equipment and with high exercise effectiveness [14]. It is an aerobic exercise to increase muscle endurance by sequentially performing 12 types of dynamic and static exercise items [30] in the cycle of 30 seconds of exercise and 10 seconds of rest.

There are 12 exercises in 7-minute HICT: jumping jacks, wall sits, push-ups, abdominal crunch, step-up onto chair, squats, triceps dip on chair, plank, high knees, lunges, push-up and rotation, and side plank.

Intermittent cyclic exercise can be divided into HICT and MICT according to exercise performance. Although HICT is more effective, both of them have significant effects on enhancing physical fitness, improving physical and mental health [13], and reducing body fat [28, 29]. However, the use of intermittent exercise models can lead to lactic acid accumulation, muscle fatigue, and decreased concentration and performance [6, 13–15, 28, 29], as well as a cyclical exercise performance and fatigue phenomenon in which exercise performance increases for 3 days and then decreases immediately the next day and then increases slowly [14]. However, because of the short time required, high efficiency, few tools, and easy operation, it is still adopted by the public [12].

### 2.2. Physical Adaptability and Body Composition

Due to changes in lifestyle behaviors, reduced exercise activities, increased sedentary or lying-down time, and high environmental risks in the community caused by COVID-19, people's willingness to go out for exercise has decreased, and university students are showing warning signs of physical adaptability, health, and blood pressure [2, 3, 7]. By using physical adaptability and body composition as the test criteria, we can obtain basic information on their current physical and mental health status.

Physical fitness can also be referred to as the body's ability to adapt or work [31]. People are physically fit if they can adapt to their daily performance, activities, and surroundings. It can be examined in terms of cardiopulmonary fitness, muscle fitness, flexibility, and body composition [32]. Blood pressure is also one indicator and a basis for predicting the performance of an individual's health and work capacity [33]. The better the physical fitness, the better the adaptability and performance [34]. It is an indicator of the basic physiological ability and health of university students [35, 36].

### 2.3. Physical and Mental Health

Physical and mental health encompasses the aspects of an individual's physical and psychological health and social adjustment [37], whereby the physical, psychological, and social levels need to achieve a state of well-being [38]. The physical and psychological status of the adolescent changes under the stress of life behavior, social circumstances [2], and the COVID-19 environment [9]. Although exercise can ameliorate these problems [8, 22], it can have negative physical and psychological effects [6, 13–16, 28, 29], and it is difficult to judge the effectiveness of improvements from appearance alone [39].

The issue of human physical and mental health has become a global public health issue [1, 2]. In addition to physical fitness and body composition tests, self-assessment is also a way to evaluate an individual's psychological perception [40, 41]. Because of its scientific approach, it is one of the best ways to self-check the current state of physical and mental health [42], and it can show how people feel about the current environment [24]. It is also judged from psychological, spiritual, and attitudinal aspects [24, 30, 43], such as anxiety, competence, enthusiasm, headache, abdominal pain, insomnia, stomach pain, eating irregularities, and suicidal thoughts [44, 45].

### 2.4. Tuina (Chinese Massage)

Tuina, also known as Chinese massage, is one of the ancient Chinese medical and healthcare methods [18]. It is performed by using upper limbs, with techniques such as pushing, rubbing, kneading, squeezing, pressing, tapping, shaking, pulling, and acupoint massage [19] to achieve the goal of patient comfort [46]. It is the crystal of wisdom from Chinese people's labor and disease care [18, 19].

Based on the techniques, contents, and the target of application, it can be used for medical, health promotion, and sports promotion purposes [18, 19, 47]. Massage is one of the techniques of Tuina. Studies have confirmed that massage can alleviate cardiovascular and visual diseases and has the effect of improving physical quality [48, 49]. It is inferred that the use of Chinese massage techniques on muscles should help to improve the fatigue state produced by intermittent exercise so that sports participants can prolong good sports performance and behavior and sustain health maintenance, so the study was conducted to verify the results.

## 3. Methods and Instruments

### 3.1. Study Framework, Design, and Positioning

After reading the literature [1–49] and referring to the results of related studies [6–29], the investigators determined the topic and experimental approach and then adopted a hybrid research method [50–54] to conduct experiments and questionnaires in succession. After obtaining data, data integration and comparison [54, 55] were conducted in a rigorous process and sequence and examined with multivariate verification [56, 57]. The research framework is shown in Figure 1.

Based on the literature mentioned above, 4 hypotheses are proposed in this study.

**Hypothesis 1 .**

(H1): The effect of the smart Chinese massage appliance has a similar influence on the physical adaptability of those who do middle- and high-intensity intermittent exercises.

**Hypothesis 2 .**

(H2): The effect of the smart Chinese massage appliance has a similar influence on the sports performance of those who do middle- and high-intensity intermittent exercises.

**Hypothesis 3 .**

(H3): The effect of the smart Chinese massage appliance has a similar influence on the body composition of those who do middle- and high-intensity intermittent exercises.

**Hypothesis 4 .**

(H4): The effect of the smart Chinese massage appliance has a similar influence on the physical and mental health of those who do middle- and high-intensity intermittent exercises.

### 3.2. Learning Procedures and Tools

Volunteers were first recruited and consent forms were signed. After screening and communication, 18 people were first accepted. Later, due to the degree of involvement and health factors, the unreadable data were eliminated and 10 subjects were finally selected as the main target for data analysis.

The questionnaire was compiled based on the literature [24, 30, 43–45], verified by three scholars, and then analyzed using SPSS 22.0 statistical software. Questions with a Cronbach's alpha value of 0.7 or higher [59] were included in the official questionnaire. The KMO value of the scale was 0.675, and Bartlett's approximate *χ*^2^ value was 195.76 with a df of 75, which was significant (*p* < 0.001) and considered suitable for the factor analysis. The explained variances were 32.95%, 23.13%, and 12.88%, respectively, and the total variance was 68.96%. After factor analysis, all questions were retained. The questionnaire consisted of 13 questions on psychological feelings (5), mental status (3), and attitude toward life and health (5). The alpha coefficients of the three scales were 0.920, 0.929, and 0.920, respectively, and the alpha coefficient of the total scale was 0.929. Based on the results of the above analysis, it was concluded that the questionnaire had good reliability, as shown in Table 1.

The experimental participants were then tested for physical adaptability, body composition [31–36], and physical and mental health [24, 30, 43–45] before the experiment. After the tests were completed, the experiment was started. The experiment was designed for 7 weeks, 5 days per week, and 1 time per day. Each time, the experiment was conducted in the following order: preparation for exercise (5 minutes), body composition test (8 minutes), experiment (7 minutes of high-intensity intermittent exercise), Chinese massage (15 minutes), data recording (5 minutes), and interview and discussion (10 minutes), totaling 50 minutes. After completing all the experimental sessions, the subjects' physical adaptability, body composition [31–36], and physical and mental health [24, 30, 43–45] were examined. Then, the participants were asked to do sit-ups (for testing their core muscle endurance), seated forward bend (for testing their flexibility), standing long jump (for testing their muscular power), and exercises for testing their cardiorespiratory endurance according to the physical fitness testing standards of the Ministry of Education of Taiwan [58], and the data on their sports performances were collected.

### 3.3. Analysis Method

A mixed-research method was used to obtain better and deeper results by multifaceted investigation and analysis [50–53]. Three research methods were used in this study. First, the experimental research method is used to design the experimental process. Then, the data on the participants' sports performances were collected according to the physical fitness testing standards of the Ministry of Education of Taiwan [59] and the 7-minute HICT (as described in the paragraph of literature review). Next, the quantitative research was carried out, using SPSS 26.0 statistical software to analyze data from the questionnaire, and the qualitative research was carried out by interviewing experts and respondents and obtaining their opinions. Finally, all the data were collated and analyzed using the multidimensional review method.

In terms of experimental design and tools, multifunctional cell phones, pedometers, electronic blood pressure meters, and fully automatic height and weight meters were used to examine pre- and postexperimental physical fitness, body composition items, and information on all experimental exercise processes.

The questionnaire and analysis tools were used to compile the formal questionnaire according to the literature [30, 43–45, 60], and then a web-based questionnaire platform was used to collect the opinions and SPSS 22.0 for Microsoft Windows statistical software was used to perform the basic statistical analysis and *t*-test for subsequent data comparison.

Four experts and scholars with expertise in sports training, physiology, public health, and psychological counseling were invited to review and provide their opinions based on the results of the survey.

Finally, the multivariate verification analysis method was used to integrate the information of different research subjects [56, 57], research theories, and methods and to obtain accurate knowledge and meanings by comparing the research results from multiple perspectives and multiple data [55].

### 3.4. Study Scope and Limitations

This study adopted a mixed-methods approach to examine the effects of Chinese massage on physical fitness, body composition, and physical and mental health of participants of different intermittent cycle exercises using an experimental, quantitative, and qualitative study. The subjects were Asian Chinese university students, aged 20 years. Students differed in their academic commitments, life stress, personal physical health, and athletic performance abilities. Questionnaire collection was influenced by personal and safety considerations. Due to funding, time, and manpower constraints, the study was conducted with volunteers, and the tools used were of low cost but accurate, and the questionnaires were distributed and collected using an online platform to save experimental time and cost. Therefore, due to the small sample size and the unavailability of data for validation and analysis, errors may occur. The findings of this study cannot be extended to other ethnic, national, age, or occupational backgrounds. Therefore, the above limitations are included as follow-up suggestions for other researchers to improve the results.

### 3.5. Ethical Considerations

This research was conducted using the intentional sampling method to identify the subjects combined. Therefore, all respondents agreed to provide relevant data and understood the main purpose of the study. All questionnaires and interviews were recorded and collected from anonymous and informed respondents.

## 4. Analysis of Results

### 4.1. Physical Adaptability Difference Analysis

According to the formula and literature [61], the maximum heart rate was determined to be 200. The sample data were divided into two groups of five by strength, named as high-strength (H1) and medium-strength (M) groups, for subsequent investigation.

The analysis showed that the preexperimental physical adaptations of the subjects were as follows: sit-ups (q): 28–50 (male: 30–50, female: 28–30); seated forward bend (q): 0–93 (male: 0–15 times, female: 13–93); standing long jump (cm): 138–220 (male: 180–220, female: 138–163); cardiorespiratory endurance (sec): 280–450 (male: 400–455, female: 280–330); mean speed (m/s): 2.35–3.81 (male: 2.42–3.52, female: 2.35–2.85); and maximum oxygen uptake (ml/kg/min): 35.54–48.73 (male: 35.8–48.73, female: 35.54–49.18).

After the experiment, the subjects' physical adaptability was as follows: sit-ups (q): 32–63 (male: 40–55, female: 32–63); seated forward bend (q): 12–87 (male: 12–16, female: 36–87); standing long jump (cm): 145–236 (male: 208–236, female: 146–164); cardiorespiratory endurance (sec): 220–400 (male: 390–400, female: 220–330); mean speed (m/s): 2.58–3.84 (male: 3.52–3.84, female: 3.16–3.81); and maximum oxygen uptake (ml/kg/min): 32.29–47.23 (male: 38.33–47.23, female: 32.29–43.61). All samples showed different levels of improvement, which is consistent with the literature [62, 63]. The results are shown in Table 2.

In the high-strength group, the postexperimental averages were as follows: sit-ups (q): 28–55, with a maximum of 55 (+10) for men and 35 (+5) for women; seated forward bend (q): 12–45, with a maximum of 12 (+12) for men and 45 (+5) for women; standing long jump (cm): 145–236, with a maximum of 236 (+36) for men and 146 (+7) for women; cardiorespiratory endurance (sec): 310–400, with a maximum of 390 (−65) for men and 310 (−10) for women; speed (m/s): 2.45–3.84, with a maximum of 3.75 (+0.55) for men and 2.58 (+0.1) for women; and maximum oxygen uptake (ml/kg/min): 37.8–43.49, with a maximum of 43.49 (+4.44) for men and 39.39 (+3.56) for women. It showed that male high-strength exercise participants showed greater performance improvement in sit-ups, seated forward bend, standing long jump, cardiorespiratory endurance, and speed after the experiment compared to females.

The average for the middle-strength group was as follows: sit-ups (q): 35–63, with a maximum of 42 (+12) for men and 63 (+34) for women; seated forward bend (q): 16–87, with a maximum of 16 (+1) for men and 87 (+23) for women; standing long jump (cm): 155–220, with a maximum of 220 for men (+10) and 164 for women (+5); cardiorespiratory endurance (sec): 220–390, with a maximum of 390 for men (−35) and 220 for women (−110); speed (m/s): 2.4–3.84, with a maximum of 3.84 for men (+0.35) (+0.35) and 3.81 (+1.41) for women; and maximum oxygen uptake (ml/kg/min): 32.29–47.23, with a maximum of 47.23 (−1.5) for men and 43.6 (+6.66) for women. It showed that the performance of the male participants in medium-strength exercise was higher than that of the female ones after the experiment only in the standing long jump, and the females performed better than the males in all other aspects.

A comparative analysis revealed that men in the medium-strength group showed better progress than counterparts in the high-strength group in sit-ups (+12 > +10), while men in the high-strength group performed better in seated forward bend (+12 > +1), standing long jump (+36 > +1), cardiorespiratory endurance (−65 > −35), speed (+0.55 > +0.35), and maximal oxygen uptake (+4.44 > −1.5) compared to counterparts in the medium-strength group. Women in the medium-strength group showed better progress than counterparts in the high-strength group in sit-ups (+34 > +5), seated forward bend (+23 > +5), standing long jump (+7 > +5), cardiorespiratory endurance (−110 > 10), speed (+1.14 > +0.1), and maximal oxygen uptake (+6.66 > +3.56). Therefore, for men, the medium-strength group performed better in sit-ups, while the high-strength group performed better than the medium-strength group in seated forward bend, standing long jump, cardiorespiratory endurance, and maximal oxygen uptake growth; for women, the medium-strength group performed better than the high-strength group in sit-ups, seated forward bend, speed, and maximal oxygen uptake.

### 4.2. Sports Performance Difference Analysis

As described in the experimental design, the subjects underwent intermittent cyclic exercise training containing 12 movements with an exercise cycle of 30 seconds of exercise and 10 seconds of rest for a total of 5 times a week for 7 weeks. Each exercise was followed by a Chinese massage session. This study was conducted to test the effectiveness of Chinese Tuina in restoring exercise fatigue [14, 19] and whether it could affect the exercise performance of participants with different intensities of intermittent exercise cycles [17].

It was found that both groups showed different levels of improvement in exercise performance after the experimental period, which is consistent with the literature [17].

However, it took 2 weeks (10 days) of acclimatization for the medium-strength group to show growth in performance. At the end of the training period, men's performance growth was small but stable, while women's growth was larger than men's, but it was not stable.

The relationship between exercise performance and oxygen intake of the experimental exercise items in the medium-strength group (M) was further investigated. It was found that the maximum increase of high leg was the largest, while the increase of other items was small. In addition, although the maximum oxygen intake of males increased steadily, it took 30 days to increase significantly, while the maximum oxygen intake of females also increased steadily and eventually changed, but the process was fluctuating or not obvious.

In addition, the exercise performance of the medium-strength group started to improve after the adaptation period of 1 week (5 days). At the end of the adaptation period, men showed high and stable growth in exercise performance, while women also showed growth in exercise performance, but the growth was smaller and highly stable.

The relationship between exercise performance and oxygen intake of the experimental items in the high-strength group was then investigated. It was found that the growth rate of the high leg raise was the greatest, while that of the other items was small. The growth margin only started to manifest after 5 sessions for males and after 7 sessions for females. In addition, the growth margin of exercise performance was different between male and female subjects, and the enhancement of maximal oxygen uptake was also different. In men, there was a significant increase in maximal oxygen uptake, while in women, the maximal oxygen uptake showed a small increase and was stable during the exercise period, as shown in Figure 2 (H1–H5).

Lastly, the data of different strength groups were analyzed. It was found that both groups showed significant improvement in exercise performance and maximal oxygen uptake. In the high-strength group, the growth margin was obvious with steady improvement in all exercise performance as well as steady growth in maximal oxygen uptake. In the medium-strength group, although there was an increase in performance and a change in maximal oxygen uptake which was stable for a long period of time, the changes were fluctuating and the increase in the next improvement was small.

It was also found that the squatting performance of the high-strength group increased by 5 times and decreased by 1 time after 9 training sessions. In the leg lifts, after 20 training sessions, there was an increase of 6 times and a decrease of 2 times. The maximum oxygen intake showed a steady growth of 8 times, but the growth of other items was unstable. Squat performance in the medium-strength group showed an increase of 4 times and a decrease of 1-2 times after 5 training sessions. For the leg lift, after 8 training sessions, there was an initial growth cycle of 4 increases and 1 decrease, which was gradually extended. In the 21st session, there was a steady increase in leg lift performance with 8 increases and 3 decreases. In terms of maximal oxygen uptake, there were 4 increases and 1-2 decreases in the first period, but the changes were not significant. It was only after 30 training sessions that maximal oxygen uptake started to increase. This result is similar to the literature [14] but with different changes in time and cycle.

### 4.3. Body Composition Difference Analysis

Intermittent cyclic exercise can improve health [8] in a time-saving and fast-acting manner [28, 29]. Although it produces fatigue [8, 28], with the help of massage, fatigue can be relieved [19], cardiovascular disease can be stabilized [23], and physiological status can be restored [20]. It was found that all subjects showed changes in body weight, blood pressure, and BMI, although there was no change in height. Body weight ranged from 50.1 to 64.7 kg in men and from 50.3 to 56 kg in women. Diastolic blood pressure ranged from 75 to 81 and systolic blood pressure ranged from 112 to 120 in men and diastolic blood pressure ranged from 69 to 78 and systolic blood pressure ranged from 94 to 111 in women. BMI ranged from 17.7 to 21.61 in men and from 17.71 to 21.48 in women. The results are in accordance with the literature [23] and are shown in Table 3.

The differences in body composition of different strength groups were analyzed next. In the high-strength group, the height ranged from 157 to 173, and, after the experiment, there was no change in the weights of both men and women. The mean body weight was 50.1–64.7, diastolic blood pressure was 69–79 and systolic blood pressure was 112–120, and BMI was 18.4–21.61. Although there were changes in both men and women, the changes were greater in men than in women (body weight, −1.8 > −0.3; blood pressure, D: −12 > −0.3, S: 16 > −7; BMI, −0.6 > −0.03). In the medium-strength group, height ranged from 153 to 173, and there was no change in males and females. The diastolic blood pressure was 60–81 and the systolic blood pressure was 94–116, and the BMI was 17.7–21.48. Except for systolic blood pressure (−47 > −17), the changes were more pronounced in women than in men (weight 0.2 > −0.9, diastolic blood pressure −29 > −19, and BMI −0.7 > −0.3). In addition, men in the high-strength group showed greater changes in body weight and BMI (−1.8 > −0.9, −0.6 > −0.3) than men in the medium-strength group. In contrast, women in the medium-strength group showed more significant changes in all items except height (weight +2 > +0.3, blood pressure D: −29 > −0.3, S: −17 > −7, and BMI −0.7 > −0.03) than women in the high-strength group. It can be seen that, in the high-strength group, men had greater changes in weight, blood pressure, and BMI than women but not in height. In the medium-strength group, women had more significant changes in body weight, blood pressure (diastolic blood pressure), and BMI than men, except for systolic blood pressure. In addition, men in the high-strength group showed greater changes in body weight and BMI than those in the medium-strength group, and women in the medium-strength group showed more significant changes in all items than those in the high-strength group.

### 4.4. Physical and Mental Health Perception Difference Analysis

Although intermittent cycle exercise produces fatigue, it is less time-consuming and achieves quicker results [28, 29], and applying massage afterward can stabilize cardiovascular disease conditions [23], relieve fatigue [19], and improve physical and mental health [8]. As shown in Table 3, the analysis of the pre- and postexperimental questionnaires revealed that there were significant differences (*p* < 0.05) on the issues of headache or head pressure, back pain, feeling of loss, and having suicidal thoughts. This indicates that the subjects had different feelings about headaches or head pressure, back pain, the feeling of loss, and thoughts of death before and after the experiment, and there were significant improvements after the experiment.

There was a significant difference (*p* < 0.05) between the strength groups on the issues of fear, headache or head pressure, and overeating but not others. This means that the subjects had different feelings on the issues of fear, headache or head pressure, and overeating in different strength groups, and the change was greater in the high-strength group than in the medium-strength group.

There was a significant difference only in insomnia or sleeplessness by gender (*p* < 0.05). This means that there were different feelings of insomnia or sleeplessness among the subjects of different genders, and they were more pronounced in men than in women, as shown in Table 4.

### 4.5. Discussion

#### 4.5.1. Differences in Physical Adaptability

We believe that, due to innate physiological advantages, men have better muscle composition and athletic performance than women. Women's athletic performance and intensity are not comparable to men's, but they have better willpower to learn [64], higher tolerance, and higher physical standards [65] than men. As a result, men in the high-strength group showed better performance improvement in sit-ups, seated forward bend, standing long jump, cardiorespiratory endurance, and speed after the experiment compared to women. In the medium-strength group, men only outperformed women in standing long jump, while women outperformed men in all other items.

In addition, sit-ups strengthen the core of the abdominal muscles and muscle endurance; open and closed jump can improve cardiorespiratory endurance; leg lifts and squats can increase the strength and agility of the lower limbs; stride movements can extend the lower back to help improve flexibility. However, in order to achieve the effect, it is necessary to carry out various exercises intensively and frequently within a limited period of time, which is difficult for women with inherent physiological conditions and sports performance limitations. Women have higher physical standards, are persistent, and have a strong will to learn [64]. Although they cannot engage in high-intensity exercise, they are willing to do it effectively and efficiently as long as it can improve their physical and mental health. As a result, men in the medium-strength group improved better in sit-ups than counterparts in the high-strength group, and men in the high-strength group improved better in seated forward bend, standing long jump, cardiorespiratory endurance, rate, and maximal oxygen uptake compared to counterparts in the medium-strength group. Women in the medium-strength group had better improvements in sit-ups, seated forward bend, standing long jump, cardiorespiratory endurance, speed, and maximal oxygen uptake compared to counterparts in the high-strength group.

#### 4.5.2. Exercise Performance Differences

The goal of the intermittent cycle exercise mode is to perform the cardiorespiratory aerobic exercise to train the core muscles of the lumbar and back such as the *rectus abdominis* and the oblique muscles in the lower and lateral back and to strengthen the pear-shaped muscles of the buttocks and the quadriceps and gastrocnemius muscles of the lower thighs in a short period of time [14]. Because of the high intensity of the exercise, it has a great effect on stimulating physiological adaptability and cardiorespiratory endurance [28]. Due to physiological differences, the muscle structure of males is more developed than that of females, and the BMI values of females in the sample group of this study were mostly below 20; the exercise performance of subjects of both genders increased after the experiment but with different results.

Furthermore, although the frequency of the lower limb exercise pattern was high in the experiment, it had the advantage of requiring fewer exercise tools and less space [14], which is suitable for university students who lack time and space as they only need to practice frequently for a short period of time [8, 9]. The higher the frequency and intensity of exercise, the better the effect, but it also produces faster and greater fatigue [29] and even results in a cyclical performance of exercise and fatigue [14]. Chinese massage techniques are diversified, with pressure and compression techniques helping to stimulate pain and massage and pushing techniques helping to relieve stiff muscles and promote blood circulation [48, 49], which have a great effect on relieving muscle fatigue. Because men have a higher tolerance than women, Chinese massage techniques can be used to fully apply pressure to muscle areas to relieve muscle fatigue after sports training. Although women had weaker muscles, they were more persistent in learning and more cooperative. Therefore, the exercise performance and maximum oxygen intake of both groups were significantly improved. In the high-strength group, there was a 1-2-week adaptation period, and the men experienced rapid and steady progress, while the women experienced steady but small progress, and the overall growth in exercise performance and maximal oxygen uptake was more obvious. In the medium-strength group, the change was small, and the growth margin was not significant in the next improvement, and men showed small and stable improvement, while women showed larger but unstable improvement compared to men and had different exercise cycles with different time and maintenance frequency, and their maximum oxygen intake also started to change only after different time points of training.

#### 4.5.3. Body Composition Differences

The 7-minute intermittent cycle exercise mode aims to build muscle strength in the lumbar and abdominal regions, lower back, buttocks, and lower thigh by performing cardiorespiratory aerobic exercise for short periods of time [14]. In order to achieve these results, it is necessary to perform frequent and intense exercises with a certain intensity to stimulate physiological adaptability and improve cardiorespiratory endurance [28], and the improvement of body composition of all subjects can be verified.

Men have a better innate physiological structure and exercise performance than women, and massage can promote fatigue metabolism and stabilize and reestablish exercise performance [48, 49]. Therefore, men in the high-strength group obtained long-term stable exercise results and improved physical and mental health. In women who were not able to cope with high-intensity exercise patterns due to their innate physiological disadvantages, a long-term and stable medium-intensity exercise program provided the physiologically required amount of exercise. However, for men, medium-strength exercise did not meet the physiological needs and therefore could not be used to improve the physiological status in a short period of time, resulting in no change in height of the subjects. However, there were changes in body weight, blood pressure, and BMI in the high-intensity group, and the changes in body weight, blood pressure, and BMI were greater for men than for women. In the medium-intensity group, the changes in body weight, diastolic blood pressure, and BMI were more pronounced in women than in men. In addition, men in the high-intensity group had greater changes in weight and BMI compared to counterparts in the medium-intensity group. Women in the medium-intensity group showed more significant changes compared to counterparts in the high-intensity group.

#### 4.5.4. Physical and Mental Health Perception Differences

There are already physical and mental health hazards among college students due to their lifestyle patterns, habits, and behaviors [2], and the impact of the COVID-19 epidemic [1] makes them even more serious [1–7]. Although intermittent cyclic exercise can improve physical and mental health [8, 13], it can also provide short-term, effective exercise results for university students [10]. Combination with the massage skills and techniques of Chinese Tuina can also promote blood circulation, relieve postexercise fatigue, and restore athletic performance [48, 49]. Therefore, it was verified that the subjects had different feelings of headache or head pressure, back pain, feeling of loss, and thoughts of death before and after the experiment, and the improvement was obvious after receiving the experiment.

Furthermore, exercise is effective in improving physical and mental health [8, 13] and has a stabilizing effect on mental and emotional well-being [16]. Although fatigue is easily produced [16, 29, 31], the use of sports massage can effectively relieve the fatigue phenomenon by accelerating blood circulation [48, 49] and restoring muscle strength [46]. Additionally, the higher the intensity of sports engagement, the better the physical and psychological well-being and physical fitness [13, 14]. This led to different perceptions of emotional feelings such as fear, headache or head stress, and overeating among subjects of different strength groups, and the change was greater in the high-strength group than in the medium-strength group.

Nevertheless, due to the frequent and intense nature of intermittent cyclic exercise [14], fatigue can occur even though massage can be used to reduce fatigue [29, 48, 49]. Men are more likely to accumulate fatigue because of the emphasis on personal sports performance and increased commitment to sports in a competitive environment [65], and their sleep quality is greatly affected by the stress caused by their daily routine and pattern as well as by their schoolwork. Therefore, insomnia or sleeplessness is felt differently by gender, and it is more pronounced in men than in women.

## 5. Conclusion and Suggestion

Chinese massage has significant effects on the physical fitness, sports performance, body composition, and physical and mental health of participants of intermittent cyclic exercise. In men, due to their innate physiological structure and sports performance, high-intensity exercise resulted in significant improvement in physical fitness, a high and stable increase in sports performance, and significant effects on weight, blood pressure, and BMI. Women are limited by their innate physiological structure, but they have high perseverance in learning and high physiological and appearance requirements, so high-strength exercise slightly improved their physical fitness, sports performance, and body composition. In terms of medium-strength exercise patterns, women were better than men in all physical fitness items except for standing long jump. Although women's exercise performance was unstable, their improvement of body composition was more obvious than that of men. In addition, there were 1-2-week adaptation periods for different strength groups, and the frequency and periodicity varied depending on the strength of the exercise. Headache or head pressure, back pain, feelings of loss, and thoughts of death improved significantly after the experiment, and the improvement in these perceptions was higher in the high-strength group than in the medium-intensity group. Women had better sleep quality than men. Based on the analysis results, we put forward the following suggestions:

1. About governments or schools. Make plans to integrate appropriate amount of intermittent exercises into a commonly taken course or physical education course, providing students with learning, to develop exercise habits and improve their physical and mental health.
2. About sports participants. It is suggested that men do high-intensity exercises and women do moderate-intensity exercises to achieve a significant exercise effect gradually.
3. Suggestions for future research. Due to the limitation of research scope, participants' willingness to participate, time, funding, and so forth, the number of actual participants was small. As a result, there were not enough participants and time to put a part of them into a control group. In addition, the experiment showed that there were differences in exercise performances between men and women. Therefore, it is recommended that the researchers of follow-up studies analyze the relevant data based on different genders, exercise intensities, and age groups.

## Figures and Tables

**Figure 1:** Research framework.

**Figure 2:** Growth curve analysis of experimental subjects' exercise performance.

**Table 1:** Analysis of physical and mental health questionnaire.

Facet	Issue	M	Cronbach's *α*
Psychological feelings	Increase confidence	4.13	0.919
	Feel scared	2.73	0.920
	Satisfied with work performance	3.98	0.918
	Full of enthusiasm	3.98	0.920
	Improve work efficiency	3.80	0.919

Mental status	Feeling a headache or pressure on the head	2.70	0.917
	Feel backache	3.00	0.916
	Insomnia or poor sleep	3.35	0.919

Life attitude and health	Stomach pain and indigestion	2.80	0.920
	Increase appetite	2.85	0.919
	Impatient, easy to lose temper	2.65	0.919
	Feeling lost	2.60	0.918
	Have thoughts of death	2.35	0.918

**Table 2:** Differences in physical adaptability of experimental subjects before and after the experiment.

	H1 (male)			H2 (male)			H3 (male)			H4 (female)		
	Before	After	DIFF	Before	After	DIFF	Before	After	DIFF	Before	After	DIFF
P1	43	45	+2	30	40	+10	50	55	+5	30	35	+5
P2	0	12	+12	10	12	+2	13	12	−1	40	42	+2
P3	220	232	+12	180	208	+28	200	236	+36	140	146	+6
P4	443	400	−43	455	390	−65	450	400	−50	330	310	−20
V (m/s)	3.38	3.75	+0.37	3.29	3.84	+0.55	3.33	3.75	+0.42	2.42	2.58	+0.16
VO2max	37.42	38.36	+0.94	38.33	40.33	+1	39.05	43.49	+4.44	35.8	37.8	+2

	H5 (female)			M1 (male)			M2 (female)			M3 (female)		
P1	28	32	+4	30	42	+12	30	36	+6	30	36	+6
P2	40	45	+5	15	16	+1	50	53	+3	13	36	+23
P3	138	145	+7	210	220	+10	160	164	+4	150	155	+5
P4	340	330	−10	425	390	−35	330	270	−60	330	220	−110
V (m/s)	2.35	2.45	+0.1	3.52	3.84	+0.32	2.42	2.96	+0.54	2.40	3.81	+1.41
VO2max	35.83	39.39	+3.56	48.73	47.23	−1.5	39.99	38.52	−1.47	43.60	43.61	+0.01

	M4 (female)			M5 (female)								
P1	29	35	+6	29	63	+34						
P2	93	87	−6	61	63.5	+2.5						
P3	163	163	+0	150	163	+13						
P4	301	253	−48	280	275	−5						
V (m/s)	2.65	3.16	+0.51	2.85	2.91	+0.06						
VO2max	49.18	42.52	+6.66	35.54	32.29	−3.25						

Physical adaptability-test items: P1: sit-ups, P2: seated forward bend, P3: standing long jump, P4: cardiorespiratory endurance (sec), H: high-strength, and M: medium-strength.

**Table 3:** Pre-post analysis of experimental subjects' body composition.

		H1 (male)			H2 (male)			H3 (male)			H4 (female)		
		Before	After	DIFF	Before	After	DIFF	Before	After	DIFF	Before	After	DIFF
cm		165	165	0	176	176	0	173	173	0	157	157	0
kg		49.5	50.1	+0.6	62.2	63.4	+1.2	66.5	64.7	−1.8	51.4	51.1	−0.3
kPa	D	70	75	+5	84	76	−8	90	79	−12	72	69	−0.3
	S	115	112	−3	136	120	−16	128	118	−10	114	107	−7
BMI		18.18	18.40	+0.22	20.08	20.46	+0.38	22.21	21.61	−0.6	20.76	20.73	−0.03

		H5 (female)			M1 (female)			M2 (female)			M3 (female)		
cm		157	157	0	173	173	0	163	163	0	168	168	0
kg		51.4	51.1	−0.3	62.3	61.2	−0.9	52.5	53.0	+0.5	58	56	−2
kPa	D	72	69	−0.3	100	81	−19	73	76	+3	74	78	+4
	S	114	107	−7	163	116	−47	103	111	+8	117	108	−9
BMI		20.76	20.73	−0.03	18.0	17.7	−0.3	19.75	19.94	+0.16	20.54	19.84	−0.7

		M4 (female)			M5 (female)								
cm		173	173	0	153	153	0						
kg		53.75	53	−0.75	50.5	50.3	−0.2						
kPa	D	67	73	+6	89	60	−29						
	S	114	108	−6	111	94	−17						
BMI		17.96	17.71	−0.15	21.57	21.48	−0.09						

H: high-strength; M: medium-strength.

**Table 4:** Physical and mental health perception difference analysis.

Facet	Issue	M	Capture time (before : after)	Diff- intensities (high : medium)	Gender
Psychological feelings	Increase confidence	4.13	(4.00 : 4.25)	(4.2 : 4.6)	(4.50 : 4.38)
	Feel scared	2.73	(3.20 : 2.25)	(2.6 : 3.6)^*∗*^	(5.00 : 2.63)
	Satisfied with work performance	3.98	(3.95 : 4.00)	(3.8 : 4.8)	(5.00 : 4.13)
	Full of enthusiasm	3.98	(3.95 : 4.00)	(3.8 : 4.6)	(4.50 : 4.13)
	Improve work efficiency	3.80	(3.95 : 3.65)	(3.6 : 4.6)	(4.50 : 4.00)
Mental status	Feeling a headache or pressure on the head	2.70	(3.25 : 2.15)^*∗∗∗*^	(2.8 : 3.6)^*∗∗*^	(5.00 : 2.75)
	Feel backache	3.00	(3.35 : 2.65)^*∗∗∗*^	(2.6 : 3.4)^*∗*^	(4.50 : 2.63)
	Insomnia or poor sleep	3.35	(3.55 : 3.15)	(3.2 : 3.6)^*∗*^	(5.00 : 3.00)^*∗*^
Life attitude and health	Stomach pain and indigestion	2.80	(3.25 : 2.35)	(2.8 : 3.4)	(4.50 : 2.75)
	Increase appetite	2.85	(3.30 : 2.40)	(2.4 : 3.6)^*∗*^	(5.00 : 2.50)
	Impatient, easy to lose temper	2.65	(3.20 : 2.10)	(2.4 : 3.4)	(4.50 : 2.50)
	Feeling lost	2.60	(3.25 : 1.95)^*∗*^	(2.2 : 3.6)	(5.00 : 2.38)
	Have thoughts of death	2.35	(3.10 : 1.60)^*∗∗*^	(1.6 : 3.4)	(4.50 : 2.00)

^*∗*^ *p* < 0.05, ^*∗∗*^*p* < 0.001, and ^*∗∗∗*^*p* < 0.00.

## Data Availability

No data support is provided.
